The article "Analysis of Multiple Sexual Partners among 2665 Male College Students Who Have Sexual Behaviour in Zhejiang Province, China" was published in 2022. Journal: Biomed Res Int.

# Analysis of Multiple Sexual Partners among 2665 Male College Students Who Have Sexual Behaviour in Zhejiang Province, China

**DOI:** 10.1155/2022/8006537

**Published:** 2022-08-18

**Authors:** Zhongrong Yang, Qiaoqin Ma, Weiyong Chen, Xin Zhou, Tingting Jiang, Zhihong Guo, Meihua Jin, Wanjun Chen

**Affiliations:** ^1^Huzhou Center for Disease Control and Prevention, Huzhou, 313000 Zhejiang Province, China; ^2^Department of HIV/STD Control and Prevention, Zhejiang Provincial Center for Disease Control and Prevention, Hangzhou, 310051 Zhejiang Province, China

## Abstract

**Objective:**

The objective of this study was to understand multiple sexual partners and related factors among male college students who exhibited sexual behaviour to provide a scientific basis for formulating HIV/AIDS prevention measures among college students.

**Methods:**

A stratified cluster random sampling method was conducted among 2665 male students who had sexual behaviour and were informed of the number of sexual partners from 13 colleges/universities in 11 cities in Zhejiang Province in 2018. Demographic characteristics, sexual attitudes, sexual behaviour, interventions, and related information were collected using a homemade online questionnaire. The chi-square test or univariate logistic regression in different groups was conducted for multiple sexual partners, and a logistic regression model was used in the related factor analysis.

**Results:**

A total of 2665 college students who engaged in sexual behaviour were involved in the research; among them, 485 students (18.20%) had multiple sexual partners. The results of multivariate analysis showed that the participants whose sexual orientation was homosexual (adjusted OR = 4.10, 95%CI = 2.89 − 5.80), those who had received school education about HIV testing in the previous year (adjusted OR = 1.55, 95%CI = 1.20 − 1.99), those who had accepted one-night stands (adjusted OR = 3.29, 95%CI = 2.43 − 4.47), those who had accepted commercial sex (adjusted OR = 1.89, 95%CI = 1.44 − 2.48), and those who were very confident in a condom use measure of self-efficacy (adjusted OR = 1.78, 95%CI = 1.31 − 2.41) were more likely to have multiple sexual partners. The participants who were senior students (adjusted OR = 0.51, 95%CI = 0.31 − 0.84), those whose monthly living expenses were 1001-1500 renminbi (adjusted OR = 0.69, 95%CI = 0.51 − 0.93), those who had known that “daily life and study contact cannot spread HIV” (adjusted OR = 0.59, 95%CI = 0.43 − 0.80), and those who knew that the CDC provides HIV testing (adjusted OR = 0.66, 95%CI = 0.46 − 0.95) were less likely to have multiple sexual partners.

**Conclusion:**

Multiple sexual partners were quite common among male college students who engaged in sexual behaviour. They had a separation of HIV/AIDS knowledge and action and a low rate of HIV testing. Further health education and intervention, including informing friends of strategies, are needed to guide students in correct sexual attitudes, safe sexual behaviour, and prevention of the spread of disease.

The article "Analysis of Multiple Sexual Partners among 2665 Male College Students Who Have Sexual Behaviour in Zhejiang Province, China" was published in 2022. Journal: Biomed Res Int.

## 1. Introduction

Acquired immune deficiency syndrome (AIDS) is a malignant infectious disease caused by human immunodeficiency virus (HIV) invading CD4^+^ cells, resulting in imbalance and damage to human immune function, in turn causing serious harm to the human body [1, 2]. HIV/AIDS has become a major global infectious disease and a serious global social problem affecting the world today [3, 4]. In recent years, the speed of HIV transmission in some countries, the rate of AIDS-related deaths, and the incidence of AIDS have continued to increase worldwide [5–7].

UNAIDS has proposed a plan to completely eliminate the global AIDS epidemic by 2030 [8]. However, the current global AIDS epidemic situation is still not optimistic and the proportion of young students with AIDS is increasing [9]. The AIDS epidemic among young Chinese students is relatively severe [10–12], and this group has become the key population for HIV/AIDS prevention and treatment. The main route of HIV infection in this population is sexual transmission [13]. With the widespread occurrence of premarital sex among college students, the incidence of unprotected sex has increased, as have the risk and impact of sexually transmitted diseases [14]. Simultaneously, with the emergence of internet dating apps, some students' traditional forms of making friends have changed, making it easier for this group to find sexual partners more conveniently and privately in turn increasing the risk of HIV transmission [15].

Many research surveys have shown that nearly half of the approximately 20 million cases of HIV infection each year are concentrated in 15- to 24-year-olds, who have become the key population for HIV/AIDS prevention and control and have dominated the mortality rate of infectious diseases in schools [16]. Multiple sexual partners, as one of the factors in unsafe sexual behaviour, increase the risk of HIV infection among students. Many studies from around the world have found that some students have multiple sexual partners [17, 18]. In China, 37.3% of university students had multiple sexual partners during the previous 6 months [19], and 53.2% of male college students had sexual intercourse for the first time at younger than 18 years old [20]. Therefore, there is an urgent need for HIV interventions for male college students who engage in sexual activities.

The article "Analysis of Multiple Sexual Partners among 2665 Male College Students Who Have Sexual Behaviour in Zhejiang Province, China" was published in 2022. Journal: Biomed Res Int.

Considering that having multiple sexual partner behaviours will result in a greater risk of HIV transmission among male college students who have sexual behaviours, it is very important to fully and accurately understand the related characteristics and influencing factors of male college students with multiple sexual partners to prevent the transmission of HIV in this population. However, there have been relatively few studies of the behaviour of having multiple sexual partners among male college students in Chinese universities. To close this gap, this study conducted a cross-sectional survey of male college students regarding multiple sexual partners' behaviours from October to November 2018. By discussing the current situation and the influencing factors of male college students' multiple sexual partner behaviours, it was intended to provide a scientific basis for colleges/universities to implement targeted HIV intervention work.

## 2. Materials and Methods

### 2.1. Participants

This study conducted a survey of 13 colleges/universities in 11 districts and cities in Zhejiang Province from October to November 2018, including 3 in Hangzhou and 1 in each of the other 10 cities [21]. In this study, 3 faculty members from each college/university were selected for the questionnaire survey by simple random sampling. Each selected faculty member was divided into 4 grades (from grade 1 to grade 4), and 200 students were planned for each grade. Each college/university planned to recruit 2400 participants (200 per grade × 4 grades × 3 faculties) for a total of 31,200 participants (2400 per university × 13 colleges/universities). Finally, 32,500 participants were investigated, of whom 31,674 completed the questionnaire, and the response rate for this survey was 97.46% (31,674/32,500).

A total of 31,674 students were investigated, of whom 2665 were male college/university students who self-reported sexual behaviour in the previous year and were informed of their sexual partners. This study was approved by the Ethics Committee of Zhejiang Provincial Center for Disease Control and Prevention (Batch number: 2018-036), and all respondents signed an informed consent form [21, 22].

### 2.2. Investigation Content and Methods

The investigation content and methods and the condom use efficacy measurement for this survey were consistent with our previous publication [21, 22], and the measured Cronbach alpha coefficient in this study was 0.799. Multiple sexual partner behaviour refers to having at least two sexual partners with whom one has participated in sexual behaviours in the previous year. Male college students with multiple sexual partner behaviours were defined as the multiple sexual partner group, and male college students with only sexual behaviours without multiple sexual partner behaviours were defined as the single sexual partner group. The quality control of this study was consistent with our previous publication [21].

The article "Analysis of Multiple Sexual Partners among 2665 Male College Students Who Have Sexual Behaviour in Zhejiang Province, China" was published in 2022. Journal: Biomed Res Int.

### 2.3. Statistical Analysis

SPSS software, version 21.0 (IBM, Armonk, NY, United States), was used for the data analysis [21]. Age, household registration, monthly living expenses, hometown, family relationship, grade [22], and sexual behaviour characteristics are expressed as the mean, composition ratio, or rate. The demographic characteristics of the participants were compared using the chi-square test. The number of self-reported sexual behaviours and reported sexual partners in the previous year were used as the dependent variables. The independent variables consisted of general characteristics, knowledge of prevention/treatment, sexual attitudes, characteristics of sexual behaviour, and undergoing an intervention. A univariate logistic regression method was used to analyze the influencing factors of participants' multiple sexual partner behaviours. In the results of the univariate analysis, variables with *P* < 0.1 and age were included in the model as independent variables, and multivariate logistic regression analysis was performed. Differences were considered statistically significant at *P* < 0.05 [21].

## 3. Results

### 3.1. General Demographic Characteristics of Participants

Among the 13 colleges/universities, 31,674 students were surveyed, including 14,320 male college students (45.21%). There were 2665 male college students (18.61%) who self-reported sexual behaviour and were informed of their sexual partners. Among them, there were 485 male college students with multiple sexual partners, accounting for 18.20% of the total number of sexually active male college students. The age of the participants was between 18 and 28 years old, the multiple sexual partner group's mean age was 20.08 ± 1.43 years old, and the single sexual partner group's mean age was 20.23 ± 1.40 years old. There was no significant difference in the situation of multiple sexual partners with age and family relationships among male college students who had sex, but there were significant differences in grade, household registration, source of hometown, and monthly living expenses (*P* < 0.05, Table 1).

### 3.2. Univariate Analysis of Multiple Sexual Partners among Participants

The results of the univariate analysis (Table 2) indicated that homosexual sexual orientation (crude OR = 6.48), acceptance of one-night stands (crude OR = 4.58), acceptance of commercial sex (crude OR = 3.86), acceptance of school promotion about HIV testing in the previous year (crude OR = 1.60), and a condom use self-efficacy measure of very confident (crude OR = 2.05) were risk factors for participants who had multiple sexual partners. It was also showed that knowing that “daily life and study contact cannot spread HIV” (crude OR = 0.35), knowing that “persistently using condoms correctly can reduce the risk of HIV infection and transmission” (crude OR = 0.33), actively seeking HIV counseling and testing after engaging in high-risk sexual behaviours (crude OR = 0.41), and knowing that the CDC provides HIV testing (crude OR = 0.63) were protective factors for participants who had multiple sexual partners.

The article "Analysis of Multiple Sexual Partners among 2665 Male College Students Who Have Sexual Behaviour in Zhejiang Province, China" was published in 2022. Journal: Biomed Res Int.

### 3.3. Multivariate Logistic Regression Analysis of Multiple Sexual Partners among Participants

The multivariate analysis results (Table 3) showed that the participants whose sexual orientation was homosexual (adjusted OR = 4.10, 95%CI = 2.89 − 5.80), those who had received school education about HIV testing in the previous year (adjusted OR = 1.55, 95%CI = 1.20 − 1.99), those who had accepted one-night stands (adjusted OR = 3.29, 95%CI = 2.43 − 4.47), those who had accepted commercial sex (adjusted OR = 1.89, 95%CI = 1.44 − 2.48), and those who were very confident in the condom use measure of self-efficacy (adjusted OR = 1.78, 95%CI = 1.31 − 2.41) were more likely to have multiple sexual partners. The participants who were senior students (adjusted OR = 0.51, 95%CI = 0.31 − 0.84), those whose monthly living expenses were 1001-1500 RMB (adjusted OR = 0.69, 95%CI = 0.51 − 0.93), those who knew that “daily life and study contact cannot spread HIV” (adjusted OR = 0.59, 95%CI = 0.43 − 0.80), and those who knew that the CDC provides HIV testing (adjusted OR = 0.66, 95%CI = 0.46 − 0.95) were less likely to have multiple sexual partners.

## 4. Discussion

This study showed that 18.20% of male college students with sexual behaviour had multiple sexual partners, which was less than the 37.32% incidence of multiple sexual partners in male college students reported by Zhao et al. [20]. Studies have shown that by implementing measures such as health promotion, peer education, and mobilizing students to test, their knowledge of sexual health can be improved, thereby reducing the occurrence of multiple sexual partners [23, 24]. On the basis of implementing the national requirements for HIV/AIDS prevention in colleges/universities, Zhejiang Province has continued to encourage relevant CDCs and local colleges/universities to establish a technical cooperation mechanism for prevention and control and has carried out HIV/AIDS prevention pilot projects in 13 colleges/universities.

The article "Analysis of Multiple Sexual Partners among 2665 Male College Students Who Have Sexual Behaviour in Zhejiang Province, China" was published in 2022. Journal: Biomed Res Int.

The results of this research indicated that moderate monthly living expenses (1001-1500 RMB per month) were a protective factor against the occurrence of multiple sexual partner behaviours, consistent with the results reported in Du et al.'s survey, the results of which showed that college students with high monthly consumption levels (who lived on more than 3000 RMB per month) were more likely to engage in sexual behaviours with a risk of HIV/STD infection [19]. At the same time, being a senior student was a protective factor against multiple sexual partner behaviour, which might be related to senior male college students being busy preparing for graduation and employment.

The results of this study suggested that a high degree of openness to sexual attitudes, such as acceptance of one-night stands and commercial sexual behaviours, was a risk factor for male college students with multiple sexual partners. Simultaneously, the high awareness rate of HIV/AIDS prevention knowledge was a protective factor for male college students against having multiple sexual partners. There is still room for improvement in HIV prevention and health education among Chinese students, and the earlier provision of HIV prevention education is a protective factor for college students' sexual behaviours [25]. Therefore, it is necessary to conduct sex education correctly and continue to strengthen the publicity of AIDS prevention knowledge. Being early, timely, and accurate and guiding students in establishing correct sexual concepts and attitudes have achieved the purpose of preventing the spread of AIDS and STDs.

This study showed that the sexual orientation of homosexuality was a risk factor for multiple sexual partner behaviours, which could be related to the sociocultural factors and social media use of men who have sex with men [26]. In fact, most HIV-infected people do not know their current infection status [27]. The CDC's voluntary HIV counseling and testing (VCT) is more efficient than HIV detection in medical institutions, and knowing one's HIV infection status can prompt individuals to engage in behaviours that reduce the risk of transmission and achieve the effect of preventing HIV transmission [28–30].

Knowledge of HIV/AIDS prevention plays a key role in reducing the risk of HIV infection [31]. The results of this study suggested that students who had received school publicity about HIV testing and had very confident self-efficacy in condom use in the previous year were risk factors for multiple partner behaviour, while knowing that the CDC offered HIV testing was a protective factor against having multiple sexual partners. However, only 11.59% of all sexually active male college students underwent HIV testing, suggesting that they had a separation of knowledge and action, and the detection rate was relatively low. Therefore, it is necessary to further emphasize the role of peer education and the CDC's VCT service, increase the HIV detection rate of male college students who exhibit sexual behaviours, and promote informed dating to reduce unprotected and unsafe sexual behaviours.

The article "Analysis of Multiple Sexual Partners among 2665 Male College Students Who Have Sexual Behaviour in Zhejiang Province, China" was published in 2022. Journal: Biomed Res Int.

This study has the following limitations. First, this study was a cross-sectional survey, and no causal inferences could be made regarding the influencing factors. Second, the content of this survey was self-reported by the research participants, and so there could be some bias. In addition, the questionnaire design of this study lacked influential information, such as the time of first sexual behaviour. Nonetheless, we performed a multivariate logistic regression analysis in the manuscript to reduce the effects of confounding factors in this study.

## 5. Conclusions

Multiple sexual partner behaviours are more common among male college students who engage in sexual behaviours. In addition, they have a separation of AIDS knowledge and action and a low rate of HIV testing, leading to a more severe HIV epidemic situation in this population. Therefore, it is necessary to undertake multiple measures to intervene in HIV/AIDS prevention education for college students. By actively guiding students to correct their attitudes towards sexual behaviour, establish correct sexual concepts, emphasize informed friendships, and advocate for safe sexual behaviours, the risk of HIV/STD transmission on campus can be reduced.

## Figures and Tables

**Table 1:** Demographic characteristics of participants.

Variables	Multiple sexual partner group (*n* = 485, %)	Single sexual partner group (*n* = 2180, %)	*x* ^2^	*P*
Age (years)				
18-19	162 (33.4)	640 (29.4)	3.761	0.152
20-21	250 (51.5)	1158 (53.1)		
22-28	73 (15.1)	382 (17.5)		
Grades				
Freshman	95 (19.6)	417 (19.1)	13.863	0.003
Sophomore	164 (33.8)	660 (30.3)		
Junior	168 (34.6)	689 (31.6)		
Senior	58 (12.0)	414 (19.0)		
Household registration^∗^			4.180	0.041
Other provinces	124 (25.6)	660 (30.3)		
Zhejiang Province	360 (74.4)	1518 (69.7)		
Hometown			10.210	0.001
Rural area	263 (54.2)	1353 (62.1)		
Town/city	222 (45.8)	827 (37.9)		
Monthly living expenses (RMB)			26.652	<0.001
≦1000	150 (30.9)	553 (25.4)		
1001-1500	136 (28.0)	886 (40.6)		
≧1501	199 (41.0)	741 (34.0)		
Family relationship			1.300	0.254
Harmonious	383 (79.0)	1669 (76.6)		
General/disharmonious/divorced	102 (21.0)	511 (23.4)		

^∗^There is missing data.

**Table 2:** Univariate analysis of multiple sexual partners among participants.

Variables	Multiple sexual partner group	Single sexual partner group	OR (95% CI)	*P*
	*n* (%)	*n* (%)		
Sexual orientation				
Heterosexual	368 (15.0)	2078 (85.0)	1	
Homosexual	117 (53.4)	102 (46.6)	6.48 (4.86-8.64)	<0.001
Whether daily life and study contact cannot spread HIV?				
No	117 (24.1)	219 (10.0)	1	
Yes	368 (75.9)	1961 (90.0)	0.35 (0.27-0.45)	<0.001
Whether adherence to correct condom use can reduce the risk of contracting and transmitting HIV?				
No	40 (8.2)	63 (2.9)	1	
Yes	445 (91.8)	2117 (97.1)	0.33 (0.22-0.50)	<0.001
Whether to seek HIV counseling and testing after high-risk sex?				
No	46 (9.5)	90 (4.1)	1	
Yes	439 (90.5)	2090 (95.9)	0.41 (0.28-0.60)	<0.001
Have you received school publicity about HIV testing in the last year?				
No	143 (29.5)	874 (40.1)	1	
Yes	342 (70.5)	1306 (59.9)	1.60 (1.29-1.98)	<0.001
Could you accept a one-night stand?				
No	100 (20.6)	1184 (54.3)	1	
Yes	385 (79.4)	996 (45.7)	4.58 (3.62-5.79)	<0.001
Could you accept commercial sex behaviour?				
No	203 (41.9)	1603 (73.5)	1	
Yes	282 (58.1)	577 (26.5)	3.86 (3.15-4.73)	<0.001
Have you received HIV testing services?				
No	401 (82.7)	1955 (89.7)	1	
Yes	84 (17.3)	225 (10.3)	1.82 (1.39-2.39)	<0.001
Did you know that the CDC offers HIV testing?				
No	71 (14.6)	212 (9.7)	1	
Yes	414 (85.4)	1968 (90.3)	0.63 (0.47-0.84)	0.002
Measurement of condom use self-efficacy^∗^				
No confidence	97 (20.9)	641 (30.0)	1	
Have confidence	140 (30.2)	768 (35.9)	1.21 (0.91-1.59)	0.191
Very confident	227 (48.9)	731 (34.2)	2.05 (1.58-2.66)	<0.001

^∗^There is missing data.

The article "Analysis of Multiple Sexual Partners among 2665 Male College Students Who Have Sexual Behaviour in Zhejiang Province, China" was published in 2022. Journal: Biomed Res Int.

**Table 3:** Multivariate analysis of multiple sexual partners among participants.

Variables	Multiple sexual partner group	Single sexual partner group	Adjusted OR (95% CI)	*P*
	*N* (%)	*N* (%)		
Age (years)				
18-19	162 (33.4)	640 (29.4)	1	
20-21	250 (51.5)	1158 (53.1)	1.02 (0.74-1.41)	0.888
22-28	73 (15.1)	382 (17.5)	1.27 (0.81-2.00)	0.297
Grades				
Freshman	95 (19.6)	417 (19.1)	1	
Sophomore	164 (33.8)	660 (30.3)	0.96 (0.68-1.35)	0.809
Junior	168 (34.6)	689 (31.6)	0.89 (0.59-1.34)	0.575
Senior	58 (12.0)	414 (19.0)	0.51 (0.31-0.84)	0.008
Household registration^∗^				
Other provinces	124 (25.6)	660 (30.3)	1	
Zhejiang Province	360 (74.4)	1518 (69.7)	1.08 (0.83-1.40)	0.575
Hometown				
Rural area	263 (54.2)	1353 (62.1)	1	
Town/city	222 (45.8)	827 (37.9)	1.21 (0.95-1.53)	0.128
Monthly living expenses (RMB)				
≦1000	150 (30.9)	553 (25.4)	1	
1001-1500	136 (28.0)	886 (40.6)	0.69 (0.51-0.93)	0.015
≧1501	199 (41.0)	741 (34.0)	0.97 (0.72-1.30)	0.835
Sexual orientation				
Heterosexual	368 (15.0)	2078 (85.0)	1	
Homosexual	117 (53.4)	102 (46.6)	4.10 (2.89-5.80)	<0.001
Whether daily life and study contact cannot spread HIV?				
No	117 (24.1)	219 (10.0)	1	
Yes	368 (75.9)	1961 (90.0)	0.59 (0.43-0.80)	0.001
Whether adherence to correct condom use can reduce the risk of contracting and transmitting HIV?				
No	40 (8.2)	63 (2.9)	1	
Yes	445 (91.8)	2117 (97.1)	0.57 (0.30-1.12)	0.104
Whether to seek HIV counseling and testing after high-risk sex?				
No	46 (9.5)	90 (4.1)	1	
Yes	439 (90.5)	2090 (95.9)	0.84 (0.47-1.50)	0.556
Have you received school publicity about HIV testing in the last year?				
No	143 (29.5)	874 (40.1)	1	
Yes	342 (70.5)	1306 (59.9)	1.55 (1.20-1.99)	0.001
Could you accept a one-night stand?				
No	100 (20.6)	1184 (54.3)	1	
Yes	385 (79.4)	996 (45.7)	3.29 (2.43-4.47)	<0.001
Could you accept commercial sex behaviour?				
No	203 (41.9)	1603 (73.5)	1	
Yes	282 (58.1)	577 (26.5)	1.89 (1.44-2.48)	<0.001
Have you received HIV testing services?				
No	401 (82.7)	1955 (89.7)	1	
Yes	84 (17.3)	225 (10.3)	1.37 (0.98-1.92)	0.067
Did you know that the CDC offers HIV testing?				
No	71 (14.6)	212 (9.7)	1	
Yes	414 (85.4)	1968 (90.3)	0.66 (0.46-0.95)	0.027
Measurement of condom use self-efficacy^∗^				
No confidence	97 (20.9)	641 (30.0)	1	
Have confidence	140 (30.2)	768 (35.9)	1.26 (0.91-1.73)	0.162
Very confident	227 (48.9)	731 (34.2)	1.78 (1.31-2.41)	<0.001

^∗^There is missing data.

The article "Analysis of Multiple Sexual Partners among 2665 Male College Students Who Have Sexual Behaviour in Zhejiang Province, China" was published in 2022. Journal: Biomed Res Int.

## Data Availability

The datasets generated and analyzed during the current study are available from the corresponding authors on reasonable request.

## Abbreviations

HIV: Human immunodeficiency virus
AIDS: Acquired immune deficiency syndrome
STD: Sexually transmitted disease
RMB: Renminbi
CDC: Center for Disease Control and Prevention
VCT: Voluntary HIV counseling and testing.
